The article "Efficacy of Traditional Chinese Medicine Combined with Chemotherapy in the Treatment of Gastric Cancer: A Meta-analysis" was published in 2022. Journal: Comput Math Methods Med.

# Efficacy of Traditional Chinese Medicine Combined with Chemotherapy in the Treatment of Gastric Cancer: A Meta-analysis

**DOI:** 10.1155/2022/8497084

**Published:** 2022-08-04

**Authors:** Wenxin Zhang, Yijuan Zhao, Hongbo Liu, Chunying Jing

**Affiliations:** ^1^Department of Gastroenterology, Lingshui County Hospital of Traditional Chinese Medicine, Lingshui, 572400 Hainan, China; ^2^Internal Medicine, Dongfang People's Hospital, Dongfang, 572600 Hainan, China; ^3^College of Traditional Chinese Medicine, Hainan Medical University, Haikou, 571199 Hainan, China

## Abstract

**Objective:**

Meta-analysis was conducted to explore the effects of CM combined with chemotherapy on the effective rate and survival rate of gastric cancer patients.

**Methods:**

Literature retrieval was performed in PubMed, MEDLINE, Embase, CENTRAL, and CNKI databases. The subject of the literature was to compare the efficacy of CM combined with chemotherapy and chemotherapy alone in patients with gastric cancer. According to the Cochrane manual, the risk of bias was assessed for inclusion in randomized controlled trials. The chi-square test was used for the heterogeneity test. Subgroup analysis and sensitivity analysis were used to explore the causes of heterogeneity. Funnel chart and Egger's test were used to assess publication bias.

**Results:**

This study included 761 patients with gastric cancer from 10 literatures. The effective rate of chemotherapy in the CM combined group was higher than that in the chemotherapy alone group (odds ratio (OR) = 1.96, 95% confidence interval (CI) (1.39, 2.78), *Z* = 3.81, *P* = 0.0001), and there was no heterogeneity among studies (chi^2^ = 5.68, *P* = 0.68, *I*^2^ = 0%). There was no significant publication bias among all studies (*P* > 0.05). The one-year survival rate in the CM combined group was higher than that in the chemotherapy alone group (OR = 3.25, 95% CI (1.90, 5.54), *Z* = 4.32, *P* < 0.0001). There was no heterogeneity among studies (chi^2^ = 1.04, *P* = 0.79, *I*^2^ = 0%) and no significant publication bias among studies (*P* > 0.05). The 3-year survival rate of gastric cancer patients in the traditional Chinese medicine combination group was higher than that in the chemotherapy alone group (OR = 1.71, 95% CI (1.06, 2.78), *Z* = 2.18, *P* = 0.03). There was no heterogeneity among studies (chi^2^ = 2.18, *P* = 0.54, *I*^2^ = 0%), and there was no significant publication bias (*P* > 0.05). The incidence of nausea and vomiting after chemotherapy in gastric cancer patients in the Chinese medicine combination group was lower than that in the chemotherapy alone group (OR = 0.47, 95% CI (0.34, 0.64), *Z* = 4.80, *P* < 0.00001). There was no heterogeneity among studies (chi^2^ = 8.57, *P* = 0.48, *I*^2^ = 0%), and there was no significant publication bias (*P* > 0.05).

**Conclusion:**

CM combined with chemotherapy can improve the effective rate and survival rate of gastric cancer and reduce the incidence of nausea and vomiting after chemotherapy. We recommend a large sample size, multicenter combined randomized controlled trial for validation.

## 1. Introduction

Gastric cancer is the most common malignant tumour of the digestive system and one of the leading causes of cancer-related death worldwide [1–3]. China is a high incidence area of gastric cancer, and its incidence rate and mortality rate rank at the forefront of malignant tumours [4–6]. Surgery and chemoradiotherapy are the main methods for treating gastric cancer. Still, these methods also burden patients, including stress responses, adverse reactions, and declining quality of life [7–9]. Chemotherapy may lead to nausea and vomiting, leucopenia, thrombocytopenia, mucosal inflammation, weight loss, and other adverse reactions in patients with gastric cancer [10–13]. In the comprehensive treatment of tumours, traditional Chinese medicine, with its unique advantages, plays an indispensable role in increasing curative effect by strengthening physique, improving body tolerance, improving quality of life, and reducing adverse reactions. Previous randomized controlled trials have confirmed that traditional Chinese medicine combined with chemotherapy can enhance patients' quality of life with gastric cancer. However, the sample size of these studies was small, and there was a high risk of bias. Thus, they could not provide reliable conclusions.

Previous meta-analysis and systematic reviews were limited to the effects of traditional Chinese medicine combined with chemotherapy on adverse reactions, quality of life, and hematopoietic system of patients with gastric cancer [14, 15]. Traditional Chinese medicine combined with chemotherapy can benefit patients in the above aspects. However, whether traditional Chinese medicine can improve the efficacy and survival rate of chemotherapy in patients with gastric cancer has been controversial. Some studies have pointed out that traditional Chinese medicine combined with chemotherapy can improve the 1-year, 3-year, and 5-year survival rates of patients [16]. However, some studies have pointed out that the effects of traditional Chinese medicine combined chemotherapy and chemotherapy alone on the 1-year survival rate and 2-year survival rate of patients are similar. Still, there are differences in the 3-year survival rate [17]. Some studies have pointed out that traditional Chinese medicine cannot affect the effective rate of chemotherapy for gastric cancer [18], while some studies hold the opposite view [19, 20]. Therefore, we conducted a meta-analysis to explore the effect of traditional Chinese medicine combined with chemotherapy on the efficacy and survival rate of chemotherapy, as well as the effects of adverse reactions in patients with gastric cancer.

## 2. Materials and Methods

### 2.1. Literature Download

Literature search was conducted in PubMed, MEDLINE, Embase, CENTRAL, and CNKI databases. The search terms were (Chinese medicine OR Chinese drugs) AND (gastric cancer OR stomach cancer) AND (chemotherapy). There were no restrictions on document language and publication time.

### 2.2. Literature Screening

Inclusion criteria are as follows: (1) the subjects were chemotherapy patients with gastric cancer. (2) The experimental group and control group were set up in the study. (3) The experimental group was treated with traditional Chinese medicine combined with chemotherapy, and the control group was treated with chemotherapy alone. (4) The outcome of observation included at least one of the effective rate, survival rate, or incidence of nausea and vomiting after chemotherapy. (5) The type of study was randomized controlled study.

Literature exclusion criteria are as follows: (1) repeated reports and case reports, (2) the subjects were patients with other tumours and could not distinguish patients with gastric cancer, (3) there was no control group in the study, (4) the balance of baseline data between the experimental group and the control group was poor or baseline data were not compared, and (5) the required data cannot be obtained, and the author of the literature cannot be contacted to supplement.

### 2.3. Data Extraction

Zhang and Zhao independently extracted the data information in included literature, such as author, title, publication time, research type, number of the experimental group, number of the control group, treatment efficiency, survival rate, and incidence of nausea and vomiting after chemotherapy. The missing data in the literature could be obtained by contacting the literature author. After data extraction, two researchers performed cross-checking. In case of disagreement, Liu and Jing discuss and solve it together.

### 2.4. Literature Quality Evaluation

This paper evaluated the literature quality by Zhang and Jing. Randomized controlled trials were assessed for risk of bias according to the “Risk of bias assessment tool for randomized trials” in the Cochrane Handbook. The evaluation contents included the bias in the process of randomization, the bias from the established intervention measures, the bias of missing outcome data, the bias of outcome measurement, and the bias of selective reporting results.

### 2.5. Heterogeneity Test

The chi-square test was used for the heterogeneity test. When *I*^2^ corrected by degrees of freedom was more than 50% or *p* < 0.1, it was considered that there was heterogeneity among published literatures, and a random effect model was used. Subgroup analysis and sensitivity analysis were used to explore the causes of heterogeneity. If the source of heterogeneity cannot be found, we could only describe the literature results without merging. When the *I*^2^ corrected by degrees of freedom was less than 50% and *P* ≥ 0.1, it is considered that there is no heterogeneity among the published literatures, and the fixed effect model was used.

### 2.6. Publication Bias Assessment

Funnel chart and Egger's test were used to evaluate the publication bias. *P* > 0.05 suggested no significant publication bias, and *P* < 0.05 indicated that there was a certain publication bias.

### 2.7. Statistical Method

This study used Cochrane software RevMan5.3 statistical analysis of the data. The effect quantity was statistically described by the odds ratio (OR) and 95% confidence interval (CI). Bilateral *P* < 0.05 indicates statistically significant.

## 3. Results

### 3.1. Characteristics of Included Literature

A total of 843 literatures were retrieved in the above database. According to the screening criteria, 833 literatures were excluded. 10 literatures with 761 gastric cancer patients were included in the study, including 435 patients with traditional Chinese medicine combined chemotherapy and 326 patients with chemotherapy alone. The flow chart of literature screening is shown in Figure 1. The basic information of the literature and the risk assessment of bias are shown in Tables 1 and 2.

### 3.2. Comparison of Therapeutic Effectiveness between the Traditional Chinese Medicine Combined Group and Chemotherapy Alone Group

A total of 9 studies compared the effect of traditional Chinese medicine combined with chemotherapy and chemotherapy alone on the treatment efficiency of patients with gastric cancer included in our meta-analysis. The heterogeneity test showed that there was no heterogeneity among the nine studies (chi^2^ = 5.68, *P* = 0.68, *I*^2^ = 0%). The fixed-effect model was used for consolidation. The effective rate of chemotherapy in the combination group of traditional Chinese medicine was higher than that in the chemotherapy alone group (OR = 1.96, 95% CI (1.39, 2.78), *Z* = 3.81, *P* = 0.0001), as shown in Figure 2. Funnel chart and Egger's test showed that the scatter points were approximately symmetrically distributed within the confidence interval and there was no significant publication bias (*P* > 0.05), as shown in Figure 3.

### 3.3. Comparison of 1-Year Survival Rate between the Traditional Chinese Medicine Combined Group and Chemotherapy Alone Group

A total of 4 studies compared the effects of traditional Chinese medicine combined with chemotherapy and chemotherapy alone on the 1-year survival rate of patients with gastric cancer included in our meta-analysis. The heterogeneity test showed that there was no heterogeneity among the four studies (chi^2^ = 1.04, *P* = 0.79, *I*^2^ = 0%). The fixed-effect model was used for consolidation. The 1-year survival rate of gastric cancer patients in the traditional Chinese medicine combined group was higher than that in the chemotherapy alone group (OR = 3.25, 95% CI (1.90, 5.54), *Z* = 4.32, *P* < 0.0001), as shown in Figure 4. Funnel plots and Egger's test showed that the scatter points were approximately symmetrically distributed within the confidence interval, and there was no significant publication bias (*P* > 0.05), as shown in Figure 5.

### 3.4. Comparison of 3-Year Survival Rate between the Traditional Chinese Medicine Combination Group and Chemotherapy Alone Group

A total of 4 studies comparing the effect of traditional Chinese medicine combined with chemotherapy and chemotherapy alone on the 3-year survival rate of gastric cancer patients were included in our meta-analysis. The heterogeneity test showed that there was no heterogeneity among the 4 studies (chi^2^ = 2.18, *P* = 0.54, *I*^2^ = 0%). A fixed-effect model was used for pooling. The 3-year survival rate of gastric cancer patients in the traditional Chinese medicine combination group was higher than that in the chemotherapy alone group (OR = 1.71, 95% CI (1.06, 2.78), *Z* = 2.18, *P* = 0.03), as shown in Figure 6. Funnel plots and Egger's test showed that the scatter points were approximately symmetrically distributed within the confidence interval, and there was no significant publication bias (*P* > 0.05), as shown in Figure 7.

### 3.5. Comparison of the Incidence of Nausea and Vomiting between the Traditional Chinese Medicine Combination Group and Chemotherapy Alone Group

A total of 10 studies comparing the effects of traditional Chinese medicine combined with chemotherapy and chemotherapy alone on the incidence of nausea and vomiting after chemotherapy in gastric cancer patients were included in our meta-analysis. The heterogeneity test showed that there was no heterogeneity among the 10 studies (chi^2^ = 8.57, *P* = 0.48, *I*^2^ = 0%). A fixed-effect model was used for pooling. The incidence of nausea and vomiting after chemotherapy in gastric cancer patients in the Chinese medicine combination group was lower than that in the chemotherapy alone group (OR = 0.47, 95% CI (0.34, 0.64), *Z* = 4.80, *P* < 0.00001), as shown in Figure 8. Funnel plots and Egger's test showed that the scatter points were approximately symmetrically distributed within the confidence interval, and there was no significant publication bias (*P* > 0.05), as shown in Figure 9.

## 4. Discussion

We compared traditional Chinese medicine with combined chemotherapy and chemotherapy alone by meta-analysis. The combined treatment could improve the chemotherapy efficiency and survival rate of patients with gastric cancer and reduce the incidence of nausea and vomiting. Zhu et al. [21] showed that the Fuzhengkang granule could improve the effective rate of superselective arterial chemotherapy. The incidence of adverse reactions in gastric cancer patients treated with chemotherapy combined with traditional Chinese medicine was lower than that of gastric cancer patients treated with chemotherapy alone. The half-year survival rate and 1-year survival rate of patients treated with traditional Chinese medicine combined with chemotherapy were higher, and the median survival time was longer. They suggest that traditional Chinese medicine can upregulate the expression of interleukin-2 and tumour necrosis factors-*α* and interferon-*γ* and downregulate the expression of the soluble interleukin-2 receptor in patients undergoing chemotherapy. It may explain why traditional Chinese medicine benefits patients with gastric cancer after chemotherapy. Qi et al. [19] demonstrated that traditional Chinese medicine could improve the effective rate of chemotherapy and reduce the incidence of adverse reactions in patients with lung cancer and gastric cancer. However, there was no significant difference in platelet, leukemia, and red blood cell count between the traditional Chinese medicine combined chemotherapy group and the chemotherapy alone group. Zhou et al. [22] showed that patients with gastric cancer treated with traditional Chinese medicine combined with chemotherapy had a higher remission rate, a greater stability rate, and a higher improvement rate of life quality compared with patients treated with chemotherapy alone. Traditional Chinese medicine has a protective effect on the blood system. The incidence of leukopenia was lower in patients using traditional Chinese medicine. The study also pointed out that traditional Chinese medicine can improve the activity of natural killer cells, macrophages, and lymphocytes. Liu et al. [20] suggest that traditional Chinese medicine combined with chemotherapy can reduce the incidence of metastasis and recurrence in patients with gastric cancer within one year after the operation. Traditional Chinese medicine can improve the peripheral hemogram and immune function of patients with gastric cancer. Wang et al. [18] showed no significant difference between the traditional Chinese medicine combined chemotherapy group and chemotherapy alone group in terms of chemotherapy efficiency, clinical benefit rate, and half-year survival rate. However, the Chinese medicine combined with the chemotherapy group had a higher 1-year survival rate. Traditional Chinese medicine can reduce the incidence of adverse reactions, including leucopenia, nausea and vomiting, mucosal reaction, and fatigue. Xin et al. [23] showed that traditional Chinese medicine combined with chemotherapy could improve the remission rate and stability rate of patients with gastric cancer. Compared with chemotherapy alone, chemotherapy combined with traditional Chinese medicine can improve the clinical symptoms and quality of life of patients with gastric cancer. Traditional Chinese medicine combined with chemotherapy reduced the incidence of leucopenia. Their research also pointed out that traditional Chinese medicine can improve the immune function of patients with gastric cancer and activate immune cells through immune regulatory factors. Liu et al. [24] showed that traditional Chinese medicine could improve the short-term efficacy, immune function, and coagulation function of patients with gastric cancer undergoing chemotherapy. Traditional Chinese medicine can reduce the incidence of lymphocytopenia. Zhao et al. [25] illustrated that the effective short-term rate of traditional Chinese medicine combined chemotherapy group was higher than that of the chemotherapy alone group. Traditional Chinese medicine can improve the Karnofsky scores and stabilize the weight of patients. They also pointed out that traditional Chinese medicine can reduce peripheral nerve injury and gastrointestinal reactions. Zhou et al. [16] showed that traditional Chinese medicine could enhance the immune function of patients with gastric cancer by activating lymphocytes. In terms of 1-year survival rate, 3-year survival rate, and 5-year survival rate, traditional Chinese medicine combined with chemotherapy has more advantages. Jiang et al. [17] believed that there was no significant difference between the traditional Chinese medicine combined chemotherapy group and the chemotherapy alone group in terms of 1-year survival rate and recurrence rate, 2-year survival rate, and recurrence rate. However, the 3-year survival rate of patients in the traditional Chinese medicine combined chemotherapy group was higher than that in the chemotherapy alone group. In comparison, the recurrence rate was lower than that in the chemotherapy alone group. The Karnofsky score for traditional Chinese medicine combined with the chemotherapy group was significantly higher than that of the chemotherapy alone group.

Among the literatures we included in the analysis, the research results of traditional Chinese medicine in reducing the incidence of chemotherapy-related nausea and vomiting were consistent. In addition, a previous meta-analysis [26] also confirmed that traditional Chinese medicine combined with chemotherapy could reduce the incidence of adverse events such as nausea and vomiting in patients with gastric cancer and play a positive role in improving the quality of life score of patients with gastric cancer. The weight of gastric cancer patients treated with traditional Chinese medicine combined with chemotherapy was more stable. In patients with low-grade gastric cancer, traditional Chinese medicine combined with chemotherapy could reduce the incidence of leukopenia and oral mucositis.

A previous network meta-analysis explored the optimal regimen of traditional Chinese medicine injection combined with XELOX regimen in the treatment of gastric cancer. Javanica oil emulsion and compound Kushen injection can improve chemotherapy efficacy. However, this study is only for one chemotherapy regimen, and this conclusion cannot be generalized [27].

There are some limitations to this study. The first is that the sample size included in the analysis is small, and there may be sample selection bias. Second, there were differences in TCM and chemotherapy regimens between studies, which may have affected the results. Finally, the literature included in the analysis was at high risk of bias, reducing the confidence of the conclusions.

In conclusion, traditional Chinese medicine combined with chemotherapy can improve the treatment efficiency and survival rate of patients with gastric cancer and reduce the incidence of nausea and vomiting after chemotherapy. We suggest a large sample size, multicenter randomized controlled trial for validation.

## Figures and Tables

**Figure 1:** Flowchart of literature screening.

**Figure 2:** Forest diagram: comparison of effective rates between the Chinese medicine combination group and chemotherapy alone group.

**Figure 3:** Funnel plot: comparison of effective rates between the traditional Chinese medicine combination group and chemotherapy only group.

**Figure 4:** Forest plot: comparison of 1-year survival rate between the Chinese medicine combination group and chemotherapy alone group.

**Figure 5:** Funnel plot: comparison of 1-year survival rate between the Chinese medicine combination group and chemotherapy alone group.

**Figure 6:** Forest plot: comparison of 3-year survival rate between the Chinese medicine combination group and chemotherapy alone group.

**Figure 7:** Funnel plot: comparison of 3-year survival rate between the Chinese medicine combination group and chemotherapy alone group.

**Figure 8:** Forest diagram: comparison of the incidence of nausea and vomiting in the Chinese medicine combination group and the chemotherapy alone group.

**Figure 9:** Funnel plot: comparison of the incidence of nausea and vomiting in the combination group and chemotherapy alone group.

**Table 1:** The characteristics included literature.

Author	Year	No. of patients		CM regimen
		CM+chemotherapy	Chemotherapy	
Zhu et al. [21]	2006	40	40	Fuzheng anticancer granule, per os, 60 g, twice a day
Qi et al. [19]	2019	24	24	Xiaoaiping injection, intravenous drip, once daily
Zhou et al. [22]	1999	62	37	Shenqi Fuzheng injection 250 ml, intravenous drip, once daily
Liu et al. [20]	2009	28	19	Yiqi Bushen oral liquid, per os, twice a day
Wang et al. [18]	2007	34	32	Fuzheng Hewei decoction, per os, twice a day
Xin et al. [23]	1998	99	45	Shenqi Fuzheng injection 250 ml, intravenous drip, once daily
Liu et al. [24]	2002	35	16	Guben Yiliu III, per os, twice a day
Zhao et al. [25]	2007	30	30	Shenqi Fuzheng injection 250 ml, intravenous drip, once daily
Zhou et al. [16]	1996	35	35	Fuzheng Huoxue anticancer prescription, 100-200 mg, per os, 3 times a day
Jiang et al. [17]	2011	48	48	Self-prescribed prescription, per os, once a day

CM indicates for Chinese medicine.

**Table 2:** Risk of bias assessment of included studies.

Author	Random sequence generation	Allocation concealment	Blinding of participants and personnel	Blinding of outcome assessment	Incomplete data	Selective reporting	Other bias
Zhu et al. [21]	High risk	High risk	Low risk	Uncertain	Low risk	Low risk	Low risk
Qi et al. [19]	Low risk	High risk	High risk	High risk	Low risk	High risk	Low risk
Zhou et al. [22]	Low risk	Uncertain	Low risk	High risk	Low risk	Uncertain	Uncertain
Liu et al. [20]	High risk	High risk	Uncertain	Low risk	Low risk	Low risk	Uncertain
Wang et al. [18]	High risk	Low risk	Low risk	High risk	Low risk	Uncertain	Low risk
Xin et al. [23]	High risk	Uncertain	High risk	Low risk	High risk	Low risk	Low risk
Liu et al. [24]	High risk	High risk	Uncertain	Low risk	Low risk	Low risk	Uncertain
Zhao et al. [25]	High risk	Uncertain	Low risk	High risk	Low risk	High risk	Uncertain
Zhou et al. [16]	Low risk	Uncertain	Uncertain	Low risk	Low risk	Low risk	Low risk
Jiang et al. [17]	Low risk	Uncertain	Low risk	High risk	Low risk	High risk	Low risk

## Data Availability

The data used to support the findings of this study are included within the article.
